The article "Efficacy and Safety of rCCK96-104PE38 Targeted Drug in the General Surgical Treatment of Colon Cancer" was retracted in 2024. Reasons: signs of a paper mill; suspected computer-generated content; unreliable results or conclusions; concerns about the data.

# Efficacy and Safety of rCCK96-104PE38 Targeted Drug in the General Surgical Treatment of Colon Cancer

**DOI:** 10.1155/2022/7145606

**Published:** 2022-06-08

**Authors:** Wenbin Cao, Bo Zhang, Yang Liu

**Affiliations:** North China University of Science and Technology Affiliated Hospital, Tangshan, 063000 Hebei, China

## Abstract

To evaluate the clinical efficacy and safety of the rCCK_96-104_PE38 targeted drug in patients with colon cancer in general surgery, data of 80 patients with colon cancer who were admitted to the hospital from April 2019 to July 2021 were selected and randomly divided into the treatment group and the control group, with 40 cases in each group. Patients in the treatment group were treated with the rCCK_96-104_PE38 targeted drug, and those in the control group were treated with oxaliplatin. The treatment efficiency and incidence of adverse reactions were compared between the two groups. The inverse cholecystokinin (CCK_96-104_) was fused with pseudomonas aeruginosa exotoxin (PE38 toxin) through the gene amplification technique to construct a prokaryotic expression vector. Then, the rCCK_96-104_PE38 was purified by Ni-nitrilotriacetate (Ni-NTA) affinity chromatography, and the antitumor activity of rCCK_96-104_PE38 was verified. The results showed that the amplified rCCK_96-104_PE38 sequence was correct and the pET-28a prokaryotic expression system was adopted to successfully achieve active expression. The purified recombinant protein could induce the apoptosis of colon cancer cells in vitro and inhibit tumor growth in vivo. The total effective rate in the treatment group (80%, 32/40) was higher than that in the control group (60%, 24/40) (*P* < 0.05). To sum up, the recombinant toxin rCCK_96-104_PE38 could not only specifically adsorb the colon cancer cells with high expression of CCK2R but also effectively inhibit tumor tissue growth and proliferation. Besides, the rCCK_96-104_PE38 protein had a good anticancer effect that helped effectively reduce the incidence of adverse reactions in patients, which was worthy of promoting.

## 1. Introduction

Colon cancer is one of the most common malignant tumors in China, and it is also a kind of digestive tract malignant tumor which is prone to travel to the rectum and at the junction of the rectum and sigmoid colon, accounting for the second most common gastrointestinal tumor. According to the latest data released by the *National Cancer Center*, there are 387,600 new cases of colon cancer in China in 2015, accounting for 9.87% of all malignant tumors. Colon cancer caused 187,100 deaths, accounting for 8.01% of all cancer deaths [1–3]. Most cases occur after the age of 40 years old, and the male to female ratio is 2 : 5. When more than 80% of patients are diagnosed, they are already in the middle or at an advanced stage [4]. At present, the treatment of colon cancer is mainly the surgical resection of tumor tissue.

To reduce the probability of postoperative tumor recurrence and metastasis, radiotherapy and chemotherapy are generally combined on this basis. However, the cure rate of traditional treatment is low, and patients usually suffer greatly during the continuation of the treatment process. Traditional methods combined with antineoplastic drugs can greatly improve the cure rate, among which the commonly used antineoplastic drugs for colon cancer include 5-fluorouracil (5-FU), irinotecan, oxaliplatin, and capecitabine [5–8]. In recent years, to improve the variety of antitumor drugs and reduce the toxic effects of traditional drugs, gene therapy drugs, immunotherapy drugs, and other targeted therapy drugs are gradually applied in clinical practice, which points out a new direction for the treatment of colon cancer.

Molecular targeted therapy is a treatment method that blocks tumor growth rate and spread by interfering with specific molecules of that target tumor growth and development [9]. Molecular targeted therapy can be classified into small molecule inhibitors and monoclonal antibodies. Small molecule inhibitors can enter the cells and block the specific molecular targets, and monoclonal antibodies can bind cell surfaces specifically, both of which inhibit tumor cells by inhibiting the downstream biological functions of target molecules [10, 11]. There is substantial overexpression of the cholecystokinin type 2 receptor (CCK2R) in tumor cells of the gastrointestinal tract compared with normal cells at the time of tumor emergence. Besides, overexpression is particularly prominent in some regions of colon cancer, colorectal cancer, and gastric cancer cell lines [12–14]. The cholecystokinin (CCK) secreted by intestinal mucosal cells is highly compatible with the cholecystokinin-B receptor (CCKBR), which will accumulate in large quantities around the cancerous tissues and promote the infiltration and migration of tumor cells [15].

Due to the significant difference in the number and affinity of CCK2R between colon cancer and normal tissue surface, No.96 to No.104 amino acid of the full-length CCK was intercepted. After the reverse recombination, it was combined with pseudomonas aeruginosa exotoxin (PE38) with high cytotoxicity to construct a novel recombinant immunotoxin rCCK_96-104_PE38. This process was used to obtain a molecular drug that could target and kill colon cancer cells efficiently. The recombinant toxin was synthesized by the prokaryotic expression system. A two-step Ni-nitrilotriacetate (Ni-NTA) affinity purification method was developed combined with the tobacco etch virus (rTEV) protease to rapidly obtain the recombinant protein with high purity, high activity, and no label. The targeting characteristics of colon cancer were explored through the experiments in vitro and in vivo, which laid the foundation for preclinical trials.

The paper is further organized as follows: in Section 2, materials and methods are discussed, in Section 3, results and discussion are done, and Section 4 gives us a conclusion.

## 2. Materials and Methods

### 2.1. Materials

In this section, we will further discuss the main reagents used in this research, general data, and instruments utilized for this research.

#### 2.1.1. The Main Reagents

Ex Taq DNA polymerase, Nhe I and Bam H I restriction enzymes, protein marker (low molecular weight), nucleic acid marker (DL2000), pMD-18 T kit, and T4 DNA ligase were purchased from TaKaRa Bio Inc., Japan. The gel extraction kit and plasmid microextraction kit were purchased from Axygen, America. Yeast powder and peptone were purchased from Oxoid, Britain. Kanamycin, ampicillin, isopropyl *β*-D-1-thiogalactopyranoside (IPTG), and dithiothreitol (DTT) were purchased from Shanghai Rhawn Chemical Technology Co., Ltd, China. Ni-NTA affinity chromatography medium and Tricorn 10/150 glass column were purchased from General Electric Company, Sweden.

The rTEV protease was purchased from Shanghai Yaji Biological Science and Technology Ltd., China. RPMI1640 medium powder and fetal bovine serum were purchased from Gibco Life Technologies, America. The polyvinylidene fluoride (PVDF) membrane was purchased from Millipore, America. Fluorescent secondary antibody Dylight 488 and horseradish peroxidase (HRP)-labeled goat anti-mouse IgG antibody were purchased from Shanghai Abcam Ltd., China. Monoclonal antibody 3B9 PE38 was prepared in the laboratory. Other chemical reagents were domestic analytical pure.

*(1) Plasmid, Bacterial Strain, and Cell*. The pET-28a plasmid was purchased from Novagen, Germany. The pET-rG17PE38recombinant plasmid, the competence BL21 (DE3) PLysS, the competence DH5a, and Human hepatocyte LO2 were all stored in the laboratory.

#### 2.1.2. General Data

Data of 80 patients with colon cancer who were admitted to the hospital from April 2019 to July 2021 were selected and randomly divided into the treatment group and the control group averagely. Patients in the treatment group were treated with the rCCK_96-104_PE38 targeted drug, and patients in the control group were treated with oxaliplatin. In the treatment group, there were 25 male patients and 15 female patients whose ages ranged from 40 to 78 years old, with an average age of 62.02 ± 5.36 years old. In the control group, there were 23 male patients and 17 female patients whose ages ranged from 42 to 80 years old, with an average age of 61.05 ± 5.37 years old. The differences were insignificant but comparable (*P* > 0.05). All the treatments were approved by the hospital ethics committee, and all the patients signed the informed consent.

The inclusion criteria were as follows:

1. Patients with colon cancer diagnosis criteria in the *Guideline of Standardized Diagnosis and Treatment of Colon Cancer (Trial)*.
2. Patients who met the criteria for chemotherapy
3. Patients with an expected survival of more than 3 months

The exclusion criteria were as follows:

1. Patients who had been treated with antineoplastic drugs for a short period
2. Patients with liver and kidney failure
3. Patients with blood diseases

#### 2.1.3. The Instruments

The gene amplifier was purchased from Beijing Ruiyisi Science and Technology Co., Ltd., China. The low-temperature high-speed centrifuge was purchased from Beckman Coulter, America. The JY99-IIDN ultrasonic cell disruptor was purchased from Shanghai HuXi Industry Co., Ltd., China. The HZQ-QX full-temperature oscillator was purchased from Changzhou Guowang Instrument Manufacturing Co. Ltd., China. The MicroChemi chemiluminescence imaging system was purchased from DNR Bio-Imaging Systems Ltd., Israel.

### 2.2. Methods

In this section, we will discuss amplification of rCCK_96-104_PE38 gene, primer design, PCR amplification system, construction of prokaryotic expression vector, low-temperature induced expression of recombinant toxin rCCK_96-104_PE38, Western Blot identification, rCCK_96-104_PE38 purified by Ni-NTA affinity chromatography column, rTEV enzyme excising histidine labels, lyophilized preservation measurement of tumor inhibition rate, observation index, and efficacy evaluation and treatment.

#### 2.2.1. Amplification of rCCK_96-104_PE38 Gene

The pET-rG17PE38 was constructed and preserved, and the reverse CCK_96-104_ fragment gene was fused with the PE38 gene by using the polymerase chain reaction (PCR) method. Restriction sites NHe I and BamH I were added at both ends of the fusion gene and connected to the pET-28A gene vector so that a histidine tag on the pET-28A vector could be fused with rCCK_96-104_PE38 for the subsequent separation and purification. The rTEV enzyme-specific recognition sites were inserted between the histidine tag and target protein, and the sequences other than rCCK_96-104_PE38 could be removed by cutting with the rTEV enzyme.

#### 2.2.2. Primer Design

The amplified primers of recombinant toxin rCCK_96-104_PE38 gene were purchased from Suzhou GENEWIZ Biotechnology Co., Ltd.  Table 1 showed the primer sequences.

#### 2.2.3. PCR Amplification System

The amplification system of rCCK_96-104_PE38 gene included 0.1*μ*LE_x_Taq, 2.0 *μ*L 10 × E_x_Taq buffer, 2.0 *μ*L dNTP, 1.0 *μ*L target DNA, 1.0 *μ*L primer (forward), 1.0 *μ*L primer (reverse), 1.0 *μ*L DMSO, and 11.9 *μ*L ddH_2_O, with a total of 20.0 *μ*L. The PCR amplification program included the preliminary unwinding at 94 °C for 5 min; the unwinding at 94 °C for 45 s, annealing for the 30s, amplification for 1 min, and the cycle for 3 times; and the amplification at 72 °C for 10 min.

#### 2.2.4. Construction of Prokaryotic Expression Vector

The PCR product and pET-28a plasmid were separately subjected to double enzyme digestion at a 37 °C water bath for 3 h. The dosage of the double enzyme digestion system included 0.5 *μ*L NHe I, 0.5 *μ*L BamH I, 1 *μ*L basal buffer, and 8 *μ*L plasmids, with a total of 10 *μ*L. Then, the results of double digestion were identified by 1% agarose gel electrophoresis. The target gene and vector fragments were recovered by the gel recovery kit and ligated overnight with a T4 ligase water bath at 16 °C. The pET-28a ligating system was 1 *μ*L T4 DNA ligase, 1 *μ*L 10× buffer, 2 *μ*L pET-28a, and 6 *μ*L target DNA, with a total of 10 *μ*L. Finally, the linker product was transformed into the BL21 (DE3) PLysS receptor cells.

#### 2.2.5. Low-Temperature Induced Expression of Recombinant Toxin rCCK_96-104_PE38

The recombinant strain pET28a-rCCK_96-104_PE38 was thawed and added to a 10 mL LB medium (Kana 50 ng/mL) in a ratio of 1 : 100. The strain was placed in the incubator overnight at 37 °C and resuscitated by shaking. Then, it was transferred to another 10 mL fresh LB medium and shaken for 1.5 h at 37 °C. 1 mM isopropyl-*β*-d-thiogalactoside (IPTG) was added and shaken for 6 h. The fermented liquid was collected by the centrifuge at 4 °C and 10,000 g/min for 15 min, and the supernatant liquid was discarded. The precipitate was suspended with phosphate buffer solution (PBS) and washed twice. The ultrasonic cell disruptor was used. The total ultrasonic time was 30 min, the power was 380 W, the working time was 1 s, and the interval time was 4 s. The solution was cleared by ultrasound waves and centrifugation was done at 4 °C and 10,000 g/min for 2 h. Part of the supernatant and inclusion body samples were collected and analyzed by the 10% sodium dodecyl sulfate-polyacrylamide gel electrophoresis (SDS-PAGE) gel electrophoresis.

#### 2.2.6. Western Blot Identification

SDS-PAGE gel electrophoresis was performed on the induced protein samples of rCCK_96-104_PE38 recombinant and pET-28a blank plasmid. Subsequently, the proteins on the gel were transferred to the PVDF membrane by the electroporation instrument and sealed overnight at 4 °C with 5% skim milk powder. The confining liquid was discarded and washed 3 times with TBST (20 mM Tris-HCL, 0.15 M NaCl, 10% Tween-20). The prepared monoclonal antibody 3B9 of 2,000 times diluted PE38 was added, incubated at 37 °C for 1 h, and washed by TBST 3 times. The 4,000 times diluted HRP-labelled goat anti-mouse IgG antibody was added, incubated at 37 °C for 1 h, and washed by TBST 5 times. The ECL chemiluminescence chromogenic solution was added. It was incubated for 1 min at room temperature without light, and the image was presented by using the MicroChemi chemiluminescence imaging system.

#### 2.2.7. rCCK_96-104_PE38 Purified by Ni-NTA Affinity Chromatography Column

Induced expression was performed according to the optimized fermentation conditions, and the bacterial solution was centrifuged at a low temperature of 4°C and a high speed of 10,000 r for 15 min. The supernatant liquid was discarded, and the PBS was added for re-suspension. The supernatant liquid was removed and cleaned twice. 15 mL PBS (containing 1 mg/mL lysozyme) was added to each 1 g of recombinant bacteria for re-suspension. The thallus was broken by the ultrasonic cell disruptor. The total time was 30 min, the power was 380 W, the working time was 1 s, and the interval was 4 s. After ultrasonic disruption, the centrifugation was at a low temperature of 4 °C and a high speed of 10,000 r for 1 h. After the sediment was discarded, the supernatant was filtered with a 0.22 *μ*m filter and stored at 4 °C for a short time.

Firstly, the chromatographic column was connected. The Ni-NTA affinity chromatography column was fully balanced with the 5-10 column volumes of Ni-NTA affinity chromatography equilibrium Buffer A (50 mmol/L Tris-HCI, 0.5 mol/L NaCl, 10 mmol/L imidazoles, 10% glycerol, pH 7.0). The ultrasonic supernatant was injected into the chromatographic column-loading valve, and the sample was loaded at a flow rate of 1 mL/min. Then, 5 column volumes were eluted with the balanced buffer solution, and the peak of flow was collected. The Ni-NTA affinity chromatography elution buffer B (50 mmol/L TrIS-HCl, 0.5 mol/L NaCl, 500 mmol/L imidazole, 10% glycerol, pH 7.0) was used to adjust the concentration of the mixture to 50 mM, 100 mM, 150 mM, 200 mM, 250 mM, 300 mM, 350 mM, 400 mM, 450 mM, and 500 mM. The eluents were collected and analyzed by the 10% SDS-PAGE gel electrophoresis.

#### 2.2.8. rTEV Enzyme Excising Histidine Labels

As an anticancer drug, the recombinant toxin was characterized by high activity, low immunogenicity, and safety. Hence, the redundant sequences of a non-rCCK_96-104_PE38KDEL gene such as the h6-histidine label needed to be removed in this experiment. When the expression vector was established, the specific restriction cutting site of the rTEV enzyme was designed. After the first purification by the Ni-NTA affinity chromatography column, the recovered protein solution was desalted by dialysis and cleaved by adding the rTEV enzyme. The results were analyzed by the 10% SDS-PAGE gel electrophoresis. According to the characteristic of rTEV with hexamethyl-histidine label, the rTEV was removed by the Ni-NTA affinity chromatography, and the purity of the target protein was over 95%.

#### 2.2.9. Lyophilized Preservation

The lyophilized protectant included 5% maltose, glucose, sucrose, and mannitol. The purified recombinant protein was freeze-dried and preserved (4 °C). In the first, second, third, and fourth weeks after the lyophilization, the appropriate amount of normal saline was used for resuspension. Subsequently, it was added to the hematopoietic cell transplant (HCT) 116 medium until the final concentration of rCCK_96-104_PE38 reached 2,000 ng/mL. CCK-8 apoptosis detection kit was adopted for the determination of the tumor inhibition rate. The lyophilized recombinant toxin proteins were stored at 4 °C, -20 °C, and -80 °C. During the first, second, third, and fourth weeks after the lyophilization, the recombinant toxin proteins were suspended with normal saline. It was added to the HCT116 medium until the final concentration of rCCK_96-104_PE38 reached 2,000 ng/mL. CCK-8 apoptosis detection kit was used to determine the tumor inhibition rate.

#### 2.2.10. Measurement of Tumor Inhibition Rate

HCT116 tumor cells in the good growth state were digested by trypsin and counted with a cell counting plate. About 5 × 10^3^ cells/pore were laid in a 96-pore cell culture plate and incubated in a CO_2_ incubator at 37 °C for 4 h. After the cell adhesion, the rCCK_96-104_PE38KDEL recombinant protein with a final concentration of 2,000 ng/mL was added, and the cells were incubated in an incubator at 37 °C. After 42 h, cell morphological changes and the number of viable cells were observed and recorded on time. The colon cancer cell line HCT116 at the logarithmic growth stage was counted, which were laid in a 96-pore culture plate with about 5 × 10^3^ cells/pore. The recombinant protein rCCK_96-104_PE38 of different concentrations was added, with 5 control pores for each concentration, and it was incubated in the incubator at 37 °C. The tumor inhibition rate was measured by the CCK-8 kit 48 h later.

#### 2.2.11. Observation Index and Efficacy Evaluation

The total effective rate and incidence of adverse reactions were compared between the two groups after clinical treatment. According to the *RECIST- Efficacy Evaluation Criteria for Solid Tumors (version 1.1)* [16], the efficacy was evaluated. Complete response (CR) referred to the complete disappearance of a patient's tumor lesion. Partial response (PR) referred to a reduction in tumor volume of more than 50% that lasts longer than 1 month. Stable disease (SD) referred that the patient's condition was relatively stable, and the tumor volume was reduced between 25% and 50%. Progression disease (PD) referred to a reduction in tumor volume of less than 25%. Equation (1) shows how the total response rate is calculated:

(1) $$\begin{array}{c} Effective\;rate\;\text{of }treatment=\text{CR }rate+\text{PR }rate+\text{SD }rate. \end{array}$$

*(1) Treatment*. Patients in the treatment group were treated with the targeted drug rCCK_96-104_PE38, and the dosage was calculated according to the patient's body surface area. The dosage was 130 mg/m^2^, which was mixed with a 500 mL glucose injection at a concentration of 5%, and the treatment was performed once every three weeks. The treatment lasted for 2 weeks as a course, and the continuous treatment lasted for 3 months.

Patients in the control group were treated with oxaliplatin (Approval number: H20093811, Hangzhou Zhongmei Huadong Pharmaceutical Co., Ltd.). The treatment method, course, and time in the control group were similar to those in the treatment group.

## 3. Results and Discussion

In this section, we will discuss the results of PCR amplification product identification and expression vector construction, expression and identification of recombinant toxin rCCK_96-104_PE38, purification of rCCK_96-104_PE38 by Ni-NTA affinity chromatography, selection of lyophilized protectant and temperature, immunofluorescence detection of rCCK_96-104_PE38 on target cells, results of cell apoptosis detection, inhibition curves of tumor cell growth, tumor-suppressive effect in vivo, comparison of treatment effects between two groups, and comparison of the incidence of adverse reactions between two groups in detail.

### 3.1. Results of PCR Amplification Product Identification and Expression Vector Construction

According to the 1% agarose gel electrophoresis, there was a bright single band at 1,700 bp of the amplified product of rCCK_96-104_PE38, which was consistent with the design size of 1670 bases (Figure 1(a)). Double digestion of plasmids from cloned strains was implemented by the plasmid microextraction kit. After the transformation into BL21, the monoclonal antibody was selected. The PCR identification results showed that the expression vector of the rCCK_96-104_PE38 gene was successfully constructed in this process. (Figure 1(b)).

### 3.2. Expression and Identification of Recombinant Toxin rCCK_96-104_PE38

The recombinant strain pET28a-rCCK_96-104_PE38 was induced by IPTG, and the protein was identified by 10% SDS-PAGE gel electrophoresis. At 36 kDa, there was one more protein band than the blank control BL21 (DE3) PLysS (pET28a), which was consistent with the design of this experiment (Figure 2(a)). The Western Blot analysis showed that the specific binding protein bands in the uninduced control were very thin, while the protein products induced by IPTG showed a protein band of about 35 kDa, which was consistent with the expectation of the researcher (Figure 2(b)).

Recombinant immunotoxin was an artificial protein that combined a guidance ligand and a toxin ligand. Recombinant immunotoxins could be classified into the natural ligands fusing specific receptors and the fusing antibodies or single-chain antibodies according to the different target molecules [17, 18]. The problem with monoclonal antibodies was that their large molecular weight increased the immunogenicity of the recombinant toxin. Besides, the molecular weight was too large for the recombinant toxin molecules to penetrate blood vessels and enter the tumor tissue cells. The use of a small protein molecule from the body as a guide ligand had no immunogenicity for the patient, and the small molecular weight was conducive to the direct targeting of drugs into tumor cells. The recombinant immunotoxin rCCK_96-104_PE38 was constructed by using CCK as the guidance ligand of the recombinant toxin under the high affinity of tumor cells in CCK and its receptor CCK2R. It had a specific targeting effect on colon cancer tumor cells.

### 3.3. Purification of rCCK_96-104_PE38 by Ni-NTA Affinity Chromatography

It was purified by the NI-NTA affinity chromatography column. The expressed recombinant protein had six histidine labels, and the gradient elution was performed through the ÄKTA purifier100TM purification system. According to the SDS-PAGE gel electrophoresis analysis, the recombinant protein rCCK_96-104_PE38 eluate was obtained at imidazole concentrations of 50 mM, 100 mM, 150 mM, 200 mM, 250 mM, 300 mM, 350 mM, 400 mM, and 450 mM (Figure 3).

### 3.4. Selection of Lyophilized Protectant and Temperature

The bioactivity of the lyophilized recombinant toxin rCCK_96-104_PE38 decreased rapidly at 4 °C. All lyophilized protectants had a certain effect to delay the rate of protein inactivation, among which 5% maltose had the best protective effect, while other lyophilized protectants had no obvious effects (Figure 4(a)). After the lyophilization, the recombinant toxin was stored at 4 °C, -20 °C, and -80 °C. The results reflected that the toxin activity decreased rapidly 4 weeks after the lyophilization at 4 °C. In comparison with the preservation effect at 4 °C, it had a better preservation effect at -20 °C and -80 °C, respectively. (Figure 4(b)).

Currently, renaturation is still a difficult topic to overcome. In the renaturation rate, the renaturation cycle in which denaturation in a short time after renaturation still cannot meet the expectation [19–21]. In general, methods that reduce the rate of protein synthesis not only increase the proportion of soluble protein but also make the protein activity stable and suitable for high expression. However, there are also problems of too many miscellaneous proteins and difficult purification of proteins. Based on the research conditions in the laboratory, the soluble part of recombinant protein was maintained above 50% by reducing the protein synthesis speed, expanding the soluble protein proportion, and optimizing the medium type and temperature, which met the needs of the subsequent experiment.

### 3.5. Immunofluorescence Detection of rCCK_96-104_PE38 on Target Cells

The fluorescent secondary antibody was used to label, and the strong green fluorescence could be signally observed on the surface of colon cancer cell line HCT116 treated with recombinant toxin rCCK_96-104_PE38. Nevertheless, the fluorescence in human normal liver cells LO2 was almost invisible. Hence, the recombinant toxin rCCK_96-104_PE38 and the cells with high expression of CCK2R were observed to bound specifically as shown in Figure 5.

### 3.6. Results of Cell Apoptosis Detection

The Annexin V apoptosis detection kit was adopted to label the cells, and the results were determined by flow cytometry (Figure 6(a)). When the concentration of recombinant toxin exceeded 100 ng/mL, the cell apoptosis was obviously induced (Figure 6(b)). The apoptosis rate of HCT116 cells was measured at the concentrations of 10 ng/mL, 100 ng/mL, 500 ng/mL, and 1,000 ng/mL, respectively, within 24 h of the incubation. The results reflected that the apoptosis rate of HCT116 cells increased with the increase of recombinant toxin concentration.

### 3.7. Inhibition Curves of Tumor Cell Growth

After the rCCK_96-104_PE38 was added into the culture medium, there was rapid apoptosis of HCT116 colon cancer cells, and the apoptotic rate was like PE toxin, but there was an insignificant effect on human normal liver cells (Figure 7(a)). PE toxin could kill the HCT116 tumor cells as well as the normal LO2 liver cells, which indicated a broad spectrum of destruction to eukaryotic cells (Figure 7(b)).

PE toxin is a single chain polypeptide composed of 638 amino acids, which belongs to the two-component AB toxin family [22–25]. PE toxin is not only highly toxic but also has a very clear mechanism of toxicity on tumor cells. Moreover, there is no preexisting antibody of PE toxin in ordinary people, which is conducive to editing and modification of activity expression [26, 27]. PE38 with a size of 38 kDa could be obtained by removing amino acid residues at positions of 1-252 and 365-380 in the nonspecific domain of the PE molecule, with very low immunogenicity.

### 3.8. Tumor Suppressive Effect In Vivo

Colon cancer models were treated with the different doses of recombinant toxin rCCK_96-104_PE38 at 5 kg/mg, 10 kg/mg, and 20 kg/mg. Among them, 20 mg/kg rCCK_96-104_PE38 showed good inhibitory effect on tumor growth cells (Figure 8).

The efficacy of recombinant toxin was evaluated according to the changes in tumor volume. The inflection points of tumor volume change appeared on the 6th day of administration. The recombinant toxin at different doses (5 mg/kg, 10 mg/kg, and 20 mg/kg) could inhibit the growth of solid tumors, and the growth rate of tumor volume decreased to different degrees in each group. After 15 days of the administration, the highest concentration group (20 mg/kg) showed the obvious antitumor effect, with a tumor inhibition rate of more than 80%, and even some tumor masses could be eliminated by this technique. Consequently, the effective dose was 20 mg/kg. The results were consistent with those of Wang et al. (2020) [28].

### 3.9. Comparison of Treatment Effects between Two Groups

In Figure 9, the total effective rate in the treatment group (80%, 32/40) was higher than that in the control group (60%, 24/40) (*P* < 0.05).

Colon cancer is a common malignant tumor, with a high fatality rate, which seriously affects the safety of people's lives. Presently, the main treatment for colon cancer in China is surgical treatment. For patients with advanced colon cancer, surgery and postoperative chemotherapy can effectively prolong their life cycle [29–32]. Some patients with immune and nutritional dysfunction cannot tolerate the adverse reactions caused by surgery and postoperative chemotherapy, so it is urgent to explore new nonsurgical methods. The rCCK_96-104_PE38 is a targeted drug that binds specifically to tumor cells. The total effective rate of the treatment group (80%) was higher than that of the control group (60%), which demonstrated that the clinical efficacy of the rCCK_96-104_PE38 targeted drug in the treatment of colon cancer patients was relatively accurate and this clinical efficacy was superior to that of Xi et al. (2020) [33].

### 3.10. Comparison of Incidence of Adverse Reactions between Two Groups

The incidence of abnormal liver function, nausea and vomiting, reduced white blood cell count, oral mucositis, and sensory nerve abnormalities in the treatment group were lower than those in the control group (*P* < 0.05). There was no considerable difference in the incidence of thrombocytopenia (*P* > 0.05).  Table 2 showed the incidence of adverse reactions in the two groups.

The rCCK_96-104_PE38 had a substantial anticancer effect that was helpful in effectively reducing the incidence of abnormal liver function, nausea and vomiting, reduced white blood cell count, oral mucositis, and sensory nerve abnormalities, which was worthy of promotion.

## 4. Conclusion

The rCCK_96-104_PE38 targeted drug was reconstructed by the recombination of amino acids No.96 to No.104 on CCK with the CCK2R targeting function under the genetic engineering technology. The recombinant toxin protein contained 6 histidine tags and was purified by Ni-NTA affinity chromatography. To keep the recombinant toxin activity as much as possible, lyophilization was adopted with 5% maltose as freeze-drying protective materials and stored at -80 °C. Through the indirect immunofluorescence and flow cytometry, the recombinant toxin rCCK_96-104_PE38 could not only specifically adsorb colon cancer cells with high expression of CCK2R but also effectively inhibit the growth and proliferation of tumor tissues. Furthermore, the rCCK_96-104_PE38 protein had an ideal anticancer effect, which helped effectively reduce the incidence of adverse reactions in patients. This treatment method was worthy of promotion. Nonetheless, the deficiency of this experiment is that the combination of recombinant immunotoxin and other drugs is not compared and its clinical efficacy needs to be further explored. In conclusion, the recombinant toxin rCCK_96-104_PE38 was a potential targeted drug for colon cancer, which was expected to open a new way for the nonsurgical treatment of colon cancer.

## Figures and Tables

**Figure 1:** Electrophoretic diagrams of the recombinant toxin rCCK96-104PE38 and the double enzyme digestion agarose gel ((a) the electrophoretic diagram of rCCK96-104PE38; (b) the electrophoretic diagram of the double enzyme digestion agarose gel). Note: M: DL2000 DNA maker; 1: PCR amplification product of the rCCK96-104PE38 gene; 2: pET-28a double digestion results; 3: pMD-18T- rCCK96-104PE38 double digestion results.

**Figure 2:** Expression and identification of the recombinant toxin rCCK_96-104_PE38 in *Escherichia coli* (*E. coli*). ((a) expression of recombinant protein rCCK_96-104_PE38 in *E. coli*; (b) expression of the recombinant protein rCCK_96-104_PE38 identified by the Western Blot). Note: M: maker; 1: 0.1 mM IPTG-induced BL21 (DE3) (PET28a) empty carrier protein; 2: 0.1 mM IPTG-induced BL21 (DE3) (pET28a-rCCK_96-104_PE38) protein; 3: the *E. coli* samples without IPTG induction; 4: the *E. coli* samples induced by IPTG.

**Figure 3:** The results of Ni-NTA affinity chromatography column purified rCCK_96-104_PE38 gradient elution. Note: M: maker; 1: flowing through; 2-10: imidazole concentration elution collection solution of 50 mM, 100 mM, 150 mM, 200 mM, 250 mM, 300 mM, 350 mM, 400 mM, and 450 mM.

**Figure 4:** Cell inhibition rate under different lyophilization agents and different temperatures. ((a) cell inhibition rate of different lyophilized agents; (b) cell inhibition rate at different temperatures).

**Figure 5:** Immunofluorescence detection of rCCK_96-104_PE38 on the target cells.

**Figure 6:** Apoptosis effect of HCT116 cells by rCCK_96-104_PE38 ((a) Results of flow cytometry; (b) the number of apoptosis determined by flow cytometry; (c) apoptosis rate at different concentrations).

**Figure 7:** Inhibition curves of cell growth ((a) colon cancer cell line HCT116; (b) normal human hepatocytes LO2).

**Figure 8:** Tumor suppression in vivo of colon cancer model ((a) changes in tumor volume; (b) comparison of tumor inhibition rates at different doses of rCCK_96-104_PE38).

**Figure 9:** Comparison of treatment effect between the two groups (CR: complete response; PR: partial response; SD: stable disease). Note: Asterisks meant that compared with the treatment group, *P* < 0.05.

**Table 1:** Amplification primer of rCCK_96-104_PE38 gene.

Name	Sequences	Restriction enzyme cutting sites and special sequences
F1	5′-TTCGATTCCGGTTCAAATTCCCGGTTAACGGGTTCCGGGC-3′	/
F2	5′-GCTAATTGAAATCGCTGTATTACTAGGGCTTCGACATGTGCCCCATG-3′	Nhe I restriction enzyme cutting site
Reverse	5′-GGATAACTACAGCTATCCCTTATTCG-3′	BamH I restriction enzyme cutting site

Note: The underline indicated the Nhe I and BamH I restriction enzyme cutting sites.

**Table 2:** Comparison of the incidence of adverse reactions between the two groups.

Group	Abnormal liver function	Nausea and vomiting	Thrombocytopenia	Reduced white blood cell count	Oral mucositis	Sensory nerve abnormalities
Treatment group	5	4	11	6	4	9
Control group	14	16	12	13	12	16
*χ* ^2^	11.783	12.451	0.765	5.562	4.671	3.781
*P*	<0.05	<0.05	>0.05	<0.05	<0.05	<0.05

## Data Availability

All data included in this study are available upon request by contact with the corresponding author.
